# Application of Computer-Based Simulation Teaching Combined with PBL in Colorectal Tumor Hemorrhage

This article has been retracted.

**DOI:** 10.1155/2022/1251388

**Published:** 2022-09-09

**Authors:** Yanling Zhang, Jinyan Hu, Lingling Li, Yunpeng Zhao

**Affiliations:** ^1^Medical Oncology Department of Thoracic Cancer, Cancer Hospital of China Medical University, Liaoning Cancer Hospital and Institute, Shenyang 110042, China; ^2^Nursing Department, Chifeng Municipal Hospital, Chifeng 024000, China

## Abstract

**Objective:**

This paper aims to explore the use of computer-based simulation teaching combined with PBL in colorectal tumor bleeding.

**Methods:**

The outpatient department organized 21 nursing staffs to conduct computer simulation combined with PBL teaching, compared emergency theory and skill scores, and investigated the recognition of computer simulation teaching combined with PBL.

**Results:**

The scores of theoretical knowledge examination before training were (84.31 ± 6.39) and (92.59 ± 2.93) after training; the scores of treatment skills examination were (85.69 ± 6.15) and (95.43 ± 2.88) after training; the scores of comprehensive treatment skills before training were (76.6 ± 6.31) and (91.43 ± 2.3) after training. The results of the questionnaires showed that the nurses were more agreeable to the new teaching methods and were able to complete the tasks in strict accordance with the requirements, ultimately achieving a level of satisfaction with their progress.

**Conclusion:**

Computer simulation teaching combined with PBL can deepen general practitioners' understanding of knowledge, improve practical ability, and provide a clinical basis for improving patient resuscitation in specialized oncology hospitals.

## 1. Introduction

First-aid skills are the most important means of rescuing patients with acute illnesses, and every medical personnel should be proficient in them, but for general practitioners, they usually resuscitate less and do not have enough clinical experience [1], and training is difficult. Patients in our department are usually admitted due to sudden illness or accident, and these patients are in serious condition and develop rapidly. In order to improve the ability of our physicians to solve emergencies, our department is generally used as the focus of medical internship. Problem-based learning (PBL) is a teaching activity innovatively applied by Barrows, a professor of neurology in the United States, at McMaster University in Canada in 1967 [2]. This teaching activity is guided by constructivist theory and is centered on the person being taught, and this teaching concept has become a more popular teaching program internationally [3, 4]. Compared with the traditional lecture-based teaching model, the PBL teaching model uses the teacher as the center of the classroom and clinical problems as the motivation for nurses to learn, so that nurses can better grasp the learning content and help nurses solve various problems in learning, so that nurses can develop more advanced skills and thinking when receiving instruction, which is extremely important for the optimization of teaching activities.

It has been more than 20 years since PBL was launched in Shanghai Second Medical University and Xi'an Medical University in 1986, and some higher medical schools in China have also started to try PBL teaching.

### 1.1. Narrow Learning Community

The learning community in traditional PBL has only nurses in the classroom, so the homogeneity of group members' thinking is high, and the overall thinking level of the learning group can hardly reach a high level, which makes the design of problem solutions lack high innovation; the group of teachers is also limited to the lecturers of the course, who lack the necessary skills and motivation to participate.

### 1.2. Single Form of Problem Situation Presentation

The problems in PBL come from real, complex, and ill-structured problems in life. However, teachers in traditional PBL still use text and video to represent problem situations, which cannot give nurses an immersive feeling and make it difficult to empathize with the environment emotionally and psychologically to achieve effective transfer of knowledge.

### 1.3. High Teaching Cost

Traditional PBL requires a large number of small classrooms for group discussions, and each small classroom must be equipped with sufficient teaching tools, learning resources, and instructors. However, with the continuous expansion of Chinese universities, schools are faced with the contradiction of more nurses and fewer instructors, shortage of teaching resources such as classrooms and libraries, and tight education funding. This has led to schools implementing PBL in the form of large class discussions, where over 100 nurses are divided into small groups in a large classroom and a lead teacher leads the discussion, which is not true PBL in the true sense.

### 1.4. Simple Communication and Collaboration Channels

In traditional PBL, nurses' problem-solving process is mainly accomplished by consulting relevant textual materials and having face-to-face discussions, exchanges, and consultations with group members. Communication among nurses and between nurses and teachers is mainly focused on the classroom, but since they are at the same level of learning and have basically similar levels of thinking, there may be some difficulties in not developing nurses' critical thinking and creative thinking skills.

### 1.5. Lack of Depth and Systematic Knowledge

In teaching, if PBL is used alone, the knowledge gained gives a feeling of lack of depth and systematization, and a lot of time is wasted in group discussions. The knowledge acquired by nurses in traditional PBL teaching is sufficient for solving a selected clinical problem, but it is not broad and deep enough for mastering the systematic knowledge of a discipline, especially in some basic medical courses, because PBL breaks the integrity of basic theoretical knowledge, some contents may be missed, so it is not as deep and systematic as the theoretical learning emphasized in the traditional teaching mode, which will cause nurses to accumulate insufficient knowledge thickness of a discipline.

### 1.6. Lack of Suitable Teaching Materials

One reason for the resistance to the implementation of PBL cannot be overlooked: the lack of appropriate textbooks. Many schools implementing PBL have found that existing textbooks for basic medicine and clinical phases are not suitable for PBL and need to be rewritten, which is a challenge for both teachers and nurses with poor clinical reasoning and self-learning skills. The continuous cross-pollination between disciplines and the deepening of medical teaching reform, medical PBL is bound to change accordingly. We believe that the online virtual classroom and online virtual clinical skills center constructed by computer technology will provide a teaching platform for remote PBL and develop nurses' problem-solving skills and that telemedicine PBL will become an important development direction of PBL.

Our medical theoretical knowledge and the extensive use of high-tech top our instruments require nurses to have a more comprehensive knowledge structure and be able to skillfully apply our commonly used technologies. In recent years, the number of outpatients in our hospital has increased rapidly, and there are often difficult and critical patients from overseas. In addition to the 13 busy nursing work, inpatient nurses undertake the task of our care for outpatients. Although the number of emergency cases is small compared to that of general hospitals, the condition is aggressive, with many comorbidities, poor predictability, and serious consequences. In order to ensure the medical safety of outpatients, the outpatient department regularly organizes standardized training for nursing staff on theoretical knowledge of treatment and treatment skills and other comprehensive abilities of our care and has achieved remarkable results.

## 2. Related Work

PBL states that medical education should study not only the biological process of disease but also its connection with social groups, psychology, environment, and behavioral patterns; the purpose of education is to promote nurses to become self-motivated lifelong learners who can continuously update their knowledge.

PBL is a learning method for acquiring and synthesizing new knowledge through problem orientation [5, 6]. It uses “real problems” as a starting point for active, independent, and collaborative learning in small groups, seeking and using multiple learning resources, discovering answers to questions, and developing nurses' critical and analytical thinking skills [7, 8]. However, research has confirmed that there are special features of PBL teaching method in the practical teaching of basic clinical skills: (1) teaching of basic clinical skills contains a large amount of practical skills training, and if simple PBL teaching focuses only on theoretical problem solving, it is inevitably suspected that the theory is out of practice and cannot meet the high requirements of modern medical education standards for medical nurses' practical skills; (2) PBL teaching of basic clinical skills needs the assistance of more teaching equipment, in addition to network tools to help nurses access information, it also needs a practical teaching platform reflecting the real clinical environment; (3) the PBL teaching method for basic clinical skills has high requirements for the design of case problems, which should reflect both the basic theory and its cutting-edge advances and include clinical skills practical training projects; otherwise, it will play the role of putting the cart before the horse [9]. The PBL teaching method of basic clinical skills has higher requirements for the design of case problems, which should reflect both the basic theory and its cutting-edge advances and include clinical skills practical training items; otherwise, it will play the role of putting the cart before the horse.

Traditional PBL (or classroom PBL) emphasizes that the teacher distributes the problem (or case) to be learned to the nurses before or during the class, and the nurses collect information related to the problem through various means around the problem or (case) and analyze and organize the collected information. In the first discussion, the instructor divides the learners into learning groups, one for every five to six nurses, and gives the nurses a certain amount of time in class to discuss and divide their learning. Nurses can then look up the information again with the questions that arose from the discussion session. In the second discussion, nurses participate in the study group again with the knowledge they have developed and the problems they have identified during the learning process. For problems that exist, the nurse needs to again continue to search in depth for information about the problem, analyze, organize, and synthesize new information with old information to form a hypothesis for the final solution. At the group discussion, the whole class submits the final problem solution reached through the discussion, and finally, the teacher gives a summary and feedback.

PBL is a new teaching method that has been rapidly developing worldwide. Since its introduction by McMaster University in Canada in 1969, PBL has been used mainly in medical and vocational schools and certain other educational fields, such as life sciences, nursing, dentistry, pharmacy, veterinary medicine, public health, architecture, business, law, engineering, forestry, and sociology [10, 11].

In just a few decades, PBL has been continuously explored and introduced into practice teaching all over the world, which must have its own indelible advantages. The main manifestations are. The PBL approach is consistent with today's philosophical view of education. PBL is based on some of today's learning theories, such as constructivist theory, contextual cognitive theory, and so on. And it is also consistent with the idea of lifelong education.

Since PBL embodies certain learning principles, it (1) enhances the spontaneity of nurses' learning. The survey found that nurses who use PBL learning are more willing to participate in teaching and learning and have more positive attitudes than those in traditional teaching methods. Nurses find PBL to be a more interesting, stimulating, and enjoyable way to learn. In PBL, nurses are more likely to become spontaneous and independent learners because they are less restricted by the teacher and more independent, which provides a solid foundation for lifelong learning.

In real life, social skills are an important element in the workplace. PBL is done in a collaborative group format, which motivates group members to cooperate in solving relevant problems. Thus, the dynamic process of collaborative learning, evaluating peers, and presenting and defending one's plan to other members of the group led to significant improvements in the nurses' interpersonal skills. All nurses do not have to follow the same pattern of learning; nurses are able to learn in the way they prefer. Stimulates student autonomy in learning. Nurses must set their own learning goals and standards to test whether they are meeting expectations, which increases their sense of responsibility for their own learning and gives them a higher degree of autonomy than traditional nurses. Teachers can give timely feedback on nurses' questions and performance to help nurses plan their next steps in learning. Combining student self-assessment, peer assessment, and teacher assessment allows nurses to become more fully aware of what is wrong with their learning. We provide an environment where nurses feel competent to learn and encourage and support them to develop their own learning interests. This interactivity is not limited to the classroom but is achieved in various forms of interaction between nurses and teachers inside and outside the classroom.

Because the process from problem identification to problem-solving in PBL is a cognitive process, and the answer to the problem in PBL is not unique, there are multiple solutions, so the nurse can only find a feasible solution in various ways to achieve the set goal or the desired effect.

## 3. Methods

Nurses from Shanghai Second Medical University and Xi'an Medical University participated in the study. Before starting the medical internship in our oncology, theoretical and practical skills examinations were conducted for common diseases in our oncology such as superior vena cava compression syndrome, acute spinal cord compression, malignant pleural effusion, pericardial effusion, and malignant colorectal tumor combined with cardiopulmonary resuscitation cases, and then a case was designed by the instructor for each disease. The operation of the SimMan4000 integrated simulator from Laerdal, Norway, was used for training. The teacher created a case of superior vena cava compression syndrome, acute spinal cord compression, malignant pleural effusion, pericardial effusion, and malignant colorectal tumor combined with CPR according to the teaching content. Then, according to the problems raised by the nurses, summarized into a number of several focused problems, each student chooses a few or a problem to find information, self-study (including checking textbooks, Internet search, search library books, literature); a few days later, focused discussion, each student report what they have prepared, and then discussion, the first hypothesis to argue, when nurses encounter more difficult. When nurses encounter more difficult problems or discussions, the teacher provides the necessary guidance and conducts a mutual aid course with nurses, the last class is summarized by the teacher, and finally a theory exam is given. The computer simulation teaching uses SimMan4000 integrated simulator for CPR skills training and assessment, the problems encountered in the computer simulation training nurses can discuss again or consult the information, and get the answers and repeatedly verify on the computer simulator to come up with the correct answers. Questionnaires were distributed to nurses' evaluation of the PBL combined with computer simulation teaching method. There were 89 questionnaires distributed and 89 questionnaires were collected, with a 100% recovery rate.

1. Establish a training group with the head nurse as the leader and select senior nurses with rich experience in treatment and training as instructors. Each person undertakes several projects to organize training.
2. Formulate training plan. ①The training team will formulate outpatient treatment skills training plan and corresponding our treatment plan according to the annual nurse training plan of nursing department, combined with the characteristics of oncology outpatients and our situations that are prone to occur, such as cardiac arrest, hemorrhage (vaginal hemorrhage in cervical cancer, nasopharyngeal hemorrhage in nasopharyngeal cancer, gastrointestinal hemorrhage in liver cancer, etc.), drug allergy events, and sudden syncope, fall and suicide, etc., our treatment plan and resuscitation workflow, etc. ②The training team develops training programs and content to be focused on according to the outpatient treatment skills training plan, such as oxygen inhalation method, electric suction method, indwelling gastric tube, urinary catheterization, use of cardiac monitor and simple respirator, as well as cardiopulmonary resuscitation, cardiac defibrillation. ③ Training for nurses' comprehensive treatment ability includes the ability to identify and solve problems, our operation skills and critical care record writing ability, etc., old. Conduct training.
3. The implementation of training treatment skills training is arranged by the chief nurse, and the instructor conducts centralized training for all inpatient nurses. The training method adopts a combination of scenario simulation method and instructor operation demonstration method, and the scenario simulation method is used for key training contents, such as resuscitation of patients in cardiac arrest and hemorrhagic shock. After the training, the trainees are assessed, and the chief nurse randomly checks the assessment every month, and the assessment results are linked to the performance.
4. Effectiveness evaluation assessment is divided into three parts: theoretical knowledge of our nursing, skill operation, and comprehensive our application ability of nurses. The theoretical examination questions combined with the theoretical knowledge learned, unified questions, ≥80 points to pass; skills operation reference 55 clinical nursing technical operation scoring standards for assessment, ≥90 points to pass; nurses comprehensive our ability assessment for resuscitation of patients after the end of the assessment, including the ability of nurses to identify and solve problems, resuscitation equipment operation proficiency, oral medical advice implementation, and critical care records The assessment of writing ability is conducted, and ≥80 is qualified.

The results of clinical medicine undergraduates before and after the internship were significantly better than those before the internship, with significant differences (about 0.05), see Table 1.

In total, 98.9% of the nurses liked the teaching method combining computer simulation and PBL, 97.6% of the nurses thought that this teaching method deepened their understanding and memory and improved their practical ability, and 96.6% of the nurses thought that the teaching method combining computer simulation and PBL could cultivate both team spirit and problem-solving ability.

Before training, 16 nurses passed the treatment theory knowledge examination, with a passing rate of 76.1%, and after training, 21 nurses passed, with a passing rate of 100%; before training, 15 nurses passed the treatment skills examination, with a passing rate of 71.5%, and after training, 20 nurses passed, with a passing rate of 95.1%; before training, 16 nurses passed the treatment comprehensive ability examination, with a passing rate of 76.3%, and after training, 20 nurses passed, with a passing rate of 95.3%. After the training, 20 nurses passed the comprehensive treatment ability test, with a pass rate of 76.3%, and the pass rate was 95.3%. After the training, the nurses' treatment theory knowledge, treatment skills assessment, and treatment comprehensive ability assessment scores are significantly improved (see Table 2.

The teaching content is the interpretation of our 2015 bleeding guidelines in oncology, causes of cardiac arrest, and recognition and management of cardiac arrhythmias. The number of teaching hours were all 12 hours. The control group used the traditional teaching method, and the teacher applied the lecture method to explain and demonstrate colorectal tumor bleeding in our hospital; the experimental group used a computer simulator combined with PBL for teaching, and the computer simulator applied the SimMan4000 integrated simulator produced by Laerdal, Norway, for simulation teaching. The specific approach was as follows: each experimental group was further divided into 3 groups of 5 members each, and the teacher created a cardiac arrest scenario case according to the teaching content, discussed the information based on this case, and proposed the most likely scenario, i.e., proposed a hypothesis. Each group member reviews the information and then summarizes it to come up with a possible answer and operates and practices on the SimMan 4000 integrated simulator. Each group member acts as a nurse, doctor, and patient's family. First, the nurse finds that the patient (SimMan integrated simulator) loses consciousness, determines whether it is cardiac arrest, starts our colorectal tumor hemorrhage, and at the same time notifies the doctor, cardiac monitoring, opens the venous. One person will direct the resuscitation, two people will be responsible for chest compressions and artificial ventilation, one person will be responsible for defibrillation and one person will be responsible for intravenous drug administration, and each person will rotate different roles after proficiency. Then, there is group discussion for the teacher to review. With the help of the video, the nurses and the instructor analyzed the resuscitation process and pointed out the merits of the nurses and the aspects that needed further improvement, such as theoretical knowledge, resuscitation techniques, communication skills, and psychological status.

The teaching effectiveness was evaluated as follows:

### 3.1. Comparison of Theoretical and Skill Test Scores

Nurses in both groups were given the same difficulty of theoretical closed-book test and applied SimMan4000 integrated simulator for skill examination with computer scoring. The theoretical test scores and operational skills test scores of nurses in the experimental group for our colorectal tumor hemorrhage were significantly higher (see Table 3).

### 3.2. The Results of Questionnaire Survey for Nurses in Both Groups

After the examination, questionnaires were distributed to the nurses of both groups, which included the evaluation of the responsibility of the instructors, the approval of the teaching methods of the instructors and the evaluation of whether their theoretical and *l* clinical levels were improved. The results of the questionnaire survey are shown in Table 4.

## 4. Results

Since no universities in China have adopted multiple computer technologies to reform traditional medical PBL methods, it is difficult for us to conduct an empirical investigation study on the effects of computer technologies on reforming traditional medical PBL at this stage. In 2002, a university medical school was the first in China to establish an advanced clinical skills center using multiple technologies, including simulation and virtual technologies. At the same time, a university medical school also applied the PBL method to teaching various disciplines and achieved certain experience and effectiveness.

In the following, we will analyze the results of the questionnaire of the 2003 undergraduate clinical skills training of a university medical school and the statistical table of the questionnaire of microbiology “PBL” of a university medical school to explore the expected effect of using various computer technologies to reform the traditional medical PBL method.

The results of the 2003 undergraduate clinical skills training questionnaire at a university medical school are as follows:

The survey was conducted mainly for the participation of 2003 undergraduate nurses in clinical skills training. 104 questionnaires were distributed, 64 in the 2003 undergraduate class, and 40 in the diagnostic class. A total of 85 questionnaires were returned, and the results are shown in Tables 5–7.

The comparison of the effectiveness of teaching with or without simulation is shown in Table 8.

Figures 1–3 show the case information provided, the organization of the class, and the takeaways for the nurses.

The experimental results showed that the practical and theoretical scores of interns in the experimental group were significantly higher than those in the control group (*P* < 0.05). During the experiment, the interns in the laboratory group were satisfied with the teaching work and performed differently (*P* < 0.05)(Tables 9 and 10.

A comparison of the changes in the condition of the two groups of patients after our 0 h and 12 h is shown in Table 11.

The comparison of mortality rates between the two groups of patients at 7 and 21 days after surgery is shown in Table 12.

## 5. Discussion

Computer simulation technology has created a fully functional clinical simulation teaching environment, providing medical students with a new practical experience. Compared with traditional medical education, simulated medical education has a better training effect and has been widely used in the medical field [11, 12]. Through a large number of teaching practices, it has been proved that simulated medical training has the following advantages: (1) Cultivate teamwork spirit. The success of CPR is not achieved by one medical personnel but requires the teamwork of several medical personnel who work together and are skilled in order to achieve successful CPR and save patients' lives. This study shows that in the simulation teaching, the students learned through the CPR exercises on the computer simulator that the spirit of collaboration is important in clinical work, and the whole process of resuscitation requires mutual cooperation and cooperation in order to achieve the highest efficiency in the shortest time [13, 14]. (2) There is no risk to the patient. Due to the increasing awareness of patients' rights, the national law requires interns to inform and obtain patients' consent when treating patients, and patients are afraid that some medical operations will be harmful to them, so they oppose interns or junior doctors to perform medical operations on themselves, which makes junior doctors lack practical experience and affects the improvement of medical standards, and the medical simulation system has solved this problem well. (3) Allowing for errors and the ability to correct them quickly. When students use the simulation system, they can make mistakes, because there are no adverse consequences, they can be corrected by the instructor in a timely manner, which helps to enhance memory and avoid making similar mistakes again. (4) Can be repeatedly operated, repeated training, participants can be repeatedly operated on the medical simulation system until proficiency. (5) Can be recorded and played back, the use of video data to find their own errors in the actual operation and to discuss and evaluate. (6) Adjustable and controllable operation process. (7) Standardization of medical training and assessment.

PBL encourages students to learn actively, and the most obvious advantage of PBL compared with traditional lecture method is that it emphasizes and encourages students to learn actively, encourages students to broaden their ideas and learn creatively, and requires the integration and convergence of basic and clinical expertise in various medical disciplines [15, 16]. Students obtain and evaluate information in various ways, and in PBL, teachers can grasp the problems of students' learning by organizing students' discussion and analysis and can tailor teaching to each student's characteristics, so that the common problems can be solved more successfully [17, 18]. At the same time, after the students finish the problem-based learning, they return to the initial state of the problem, and the key contents of the teaching can be remembered and understood deeply after repeated cycles.

The combination of computer simulation teaching and PBL enhances the attractiveness of classroom teaching and students' learning ability, stimulates the enthusiasm of operation and practice, and deepens the understanding and memory of knowledge, thus completely changing the previous situation of emphasizing knowledge transfer but not ability cultivation, teacher teaching but not student participation in the teaching process [19, 20]. PBL creates “problem scenarios” and sets learning into complex and meaningful problem situations. The process of learning is to learn the scientific knowledge implied behind the problems and to develop problem-solving skills, i.e., to develop the ability to learn independently. At the same time, the ability to acquire and evaluate information and the skill to disseminate information is improved [21, 22]. Computer simulation teaching combined with PBL can cultivate students' comprehensive quality, deepen their knowledge and understanding of the original theoretical knowledge in textbooks, and train both comprehensive analysis ability and knowledge application ability, so that students can really become the discoverer and applicator of knowledge and improve their comprehensive quality. In the specific computer simulation scenario, students can exercise their teamwork and social practice [23]. The students develop practical skills and good psychological quality. Focus on inducing students to think independently, enhance the cultivation of analytical skills, and give students more opportunities for independent thinking and self-development.

This study showed that the application of computer simulation combined with PBL in CPR teaching significantly improved students' performance, and 96.8% of students liked computer simulation combined with PBL, which fully demonstrated the advantages of this teaching method [24, 25]. Seven-year students with good English, strong learning ability and high overall quality can definitely improve their academic performance and clinical skills by applying computer simulation teaching combined with PBL in teaching, and prepare to serve patients better in the future.

With the development of new surgical procedures, improved surgeon techniques and the widespread use of broad-spectrum antibiotics, the incidence of fatal bleeding has become less common, but when this complication does occur, it is often critical, clinically difficult to treat, and highly lethal. The first few minutes of treatment when bleeding occurs are critical, and correct and timely treatment by the first caregiver on the scene may save the patient's life. Therefore, it is critical for nursing staff to have the correct treatment measures in place to take accurate and effective measures to stop the bleeding and improve the success rate of resuscitation.

This study showed that the application of computer simulation teaching combined with PBL for colorectal tumor bleeding significantly improved the learning performance of nurses, and the questionnaire results showed that nurses were more agreeable to the new teaching method and were able to complete the tasks strictly in accordance with the requirements, and eventually reached a level of satisfaction with their progress. This fully reflects the advantages of computer simulation teaching combined with PBL teaching method.

In summary, PBL teaching on computer simulation system can overcome the real problem of “few practice opportunities” for medical nurses by simulating real clinical scenes and expand their clinical thinking ability through “problem-centered” heuristic teaching. The problem of low practice opportunities for medical nurses can be overcome by simulating real clinical scenarios. Through the perfect combination of teaching methods and teaching methods, it provides an important guarantee for the overall improvement of clinical practice skills of medical and nursing staff.

## Figures and Tables

**Figure 1:** Availability of case information.

**Figure 2:** Classroom organization.

**Figure 3:** Gains of the nurses.

**Table 1:** Theoretical and skill examination scores before and after the internship ($\bar{x}$ ± *s*).

Group	*n*	SVCS	Sec	Cardiopulmonary resuscitation	Practical skills
Post-apprenticeship	89	65.5 ± 8.9	71.2 ± 8.3	65.9 ± 9.6	70.5 ± 6.5
Pre-apprenticeship	89	82.3 ± 9.2	84.9 ± 7.1	82.3 ± 9.1	89.1 ± 7.9
*P*		0.018	0.027	0.012	0.008

**Table 2:** Comparison of assessment scores of 21 nurses' treatment ability before and after training (scores).

Measurement items	*n*	Treatment theory knowledge	Treatment skills assessment	Comprehensive ability of first aid
Pretraining	21	84.32 ± 6.38	85.69 ± 6.13	76.9 ± 6.28
After training	21	92.62 ± 2.90	95.42 ± 2.87	91.5 ± 2.3
*t*-value		5.408	6.590	10.096
*P*-value		<0.05	<0.05	<0.05

**Table 3:** Comparison of theoretical and skill examination scores of nurses in the experimental and control groups ($\bar{x}$ ± *s*, scores).

Group	*n*	Theoretical examination results	Practical skills
Experimental group	45	84.36 ± 7.25^*∗*^	86.20 ± 7.31^*∗∗*^
Control group	45	77.20 ± 5.24	71.35 ± 9.18^*∗∗*^

**Table 4:** Results of the questionnaire survey of 90 nurses' evaluation of the two teaching methods *n* (%).

Questionnaire items	Experimental group (*n* = 45)				Control group (*n* = 45)			
	Very satisfied	Satisfactory	General	Poor	Very satisfied	Satisfactory	General	Poor
Evaluation of teachers^*∗∗*^	24 (69.9)	9 (29.7)	0 (0)	0 (0)	9 (27.5)	22 (64.9)	5 (13.3)	0 (0)
Agreement with old and new teaching methods^*∗*^	14 (44.3)	19 (55.2)	0 (0)	0 (0)	12 (35.2)	13 (41.1)	7 (23.9)	0 (0)
Satisfaction with their own progress^*∗∗*^	17 (51.6)	16 (48.6)	0 (0)	0 (0)	5 (17.1)	14 (42.3)	13 (39.5)	0 (0)

**Table 5:** The way of gain clinical all techniques.

Evaluation content	Classroom learning and training (%)	Internet learning (%)	After-class learning, peer-to-peer practice (%)
Student evaluation results	92.93	25.89	42.36

**Table 6:** The ratio of theories study and techniques exercise.

Evaluation content	Rationality of theory and training proportion (%)	Theoretical study is less, which affects the understanding of learning content (%)	Less skill training, more optional (%)
Student evaluation results	45.89	20.00	34.11

**Table 7:** The content degree of clinical techniques training.

Evaluation content	Small class lectures, model practice (%)	SP training (%)	E-learning (%)	Other (can be specified)
Student evaluation results	74.13	27.05	2.34	

**Table 8:** The contrast of teaching effect on applying the simulated technology to teach or not.

	Trained	Untrained
Reached caecum	53%	18%
Time to caecum (min)	35	45
Pain (VAS)	6	7

**Table 9:** Comparison of assessment scores and satisfaction scores of teaching of clinical medicine interns in the two groups (points,$\bar{x}$ ± *s*).

Group	Theoretical knowledge	Hands-on
Experimental group (*n* = 35)	86.59 ± 5.64	77.68 ± 5.14
Control group (*n* = 35)	96.85 ± 5.38	93.46 ± 2.99
*T*	6.266	7.126
*P*	*P* < 0.001	*P* < 0.001

**Table 10:** Comparison of clinical medicine interns' satisfaction scores with medical teaching between the two groups.

Group	Very satisfied	Satisfactory	Dissatisfied	Total satisfaction
Experimental group (*n* = 35)	12	11	12	65.72%
Control group (*n* = 35)	14	16	5	88.56%
*x* ^2^				9.265
*P*				*P* < 0.001

**Table 11:** Comparison of changes in APACHE II scores between the two groups of patients after 0 h and 12 h of our care (score,$\bar{x}$ ± *s*).

Group	0 h	12 h
Experimental group	28.6 ± 5.5	17.4 ± 6.6
Control group	28.5 ± 5.3	23.9 ± 4.4
*t*	0.353	6.484
*P*	>0.05	<0.05

**Table 12:** Comparison of mortality rates between the two groups of patients at 7 and 21 days after surgery (cases (%)).

Group		

Experimental group	1 (1.8)	2 (3.4)
Control group	2 (3.6)	4 (6.8)
*x* ^2^	0.126	0.175
*P*	>0.05	>0.05

## Data Availability

The experimental data used to support the findings of this study can be obtained from the corresponding author upon request.
